The article "Factors Affecting Transfusion during Percutaneous Nephrolithotomy: A Retrospective Study of 665 Cases" was retracted in 2023. Reasons: signs of a paper mill; suspected computer-generated content; unreliable results or conclusions; lack of ethics approval or compliance.

# Factors Affecting Transfusion during Percutaneous Nephrolithotomy: A Retrospective Study of 665 Cases

**DOI:** 10.1155/2022/6775277

**Published:** 2022-06-06

**Authors:** Hong Zhao, Junsheng Li, Li Li, Hang Wang, Jianming Guo, Yi Miao

**Affiliations:** ^1^Department of Urology, Shanghai Xu-Hui Central Hospital, No 966, Huaihai Road, Shanghai 200032, China; ^2^Department of Urology, Zhongshan Hospital, Fudan University, No 180, Fenglin Road, Shanghai 200032, China; ^3^Department of Transfusion, Shanghai Xu-Hui Central Hospital, Shanghai 200032, China

## Abstract

**Objective:**

This study was designed to evaluate the aspects that affect transfusion following percutaneous nephrolithotomy (PCNL). *Patients and Methods*. From 2016 to 2019, 665 patients underwent PCNL for the removal of renal calculi at our center (Department of Urology, Shanghai Xu-hui Central Hospital). Complications, including hemorrhages, have been reported. Twenty-three patients (3.5%) have received a blood transfusion, and 12 (1.9%) patients were treated with hyper-selective embolization. We focused on the influencing factors related to postoperative blood transfusion. The factors analyzed were age, sex, hypertension, diabetes, serum creatinine level, preoperative hemoglobin, and the use of anticoagulants or antiplatelet medications; renal and stone factors (i.e., previous surgery, abnormal anatomy, stone side, stone burden, and stone type); and surgical features (i.e., access number, the calyx of puncture, and stone-free rate). These data were analyzed for the presence of bleeding.

**Results:**

Among individual factors, preoperative hemoglobin level (*p* < 0.001) and urinary infections (*p* < 0.001) were significantly correlated with blood transfusion. Among renal and stone factors, only a history of open surgery was significantly correlated with blood transfusion (*p* < 0.05). Stone type or stone burden did not correlate with transfusion. Furthermore, no statistically significant correlation was found between surgical features and bleeding, and a lower stone-free rate was reported for the transfusion group.

**Conclusion:**

The obtained results demonstrated that PCNL is a safer surgical procedure in a high-volume center; however, anemic conditions, infections, and history of open surgery will significantly increase the transfusion rate following PCNL.

## 1. Introduction

Since its first description in 1976 [1], percutaneous nephrolithotomy (PCNL) has been widely used for treating renal calculi. It is the gold standard therapy for treating 2-cm kidney stones [2]. Although it is an effective and safe surgical method for managing upper urinary calculi, because of the high incidence of complications, its popularity varies from place to place. Common complications include bleeding, urinary tract infection, fever, and sepsis [3]. Factors associated with an increased risk of complications include increasing patient age [3], female gender [4], long operative time [4], and comorbidities [5]. Bleeding is one of the most serious complications following PCNL. The overall transfusion rate following this surgical procedure has been reported to range from 0.8% to 17.5% in the literature [6, 7]. Moreover, 0.8% of patients require angioembolization to control intractable bleeding [8].

The article "Factors Affecting Transfusion during Percutaneous Nephrolithotomy: A Retrospective Study of 665 Cases" was retracted in 2023. Reasons: signs of a paper mill; suspected computer-generated content; unreliable results or conclusions; lack of ethics approval or compliance.

Many studies have investigated the factors associated with bleeding after PCNL. Because surgical methods differ among centers and the conditions of patients vary, the factors associated with bleeding are not unified. The trend of the transfusion rate after PCNL is lower [7]. Factors affecting bleeding during PCNL are thought to be operating time, stone load, caseload, and sheath size, among others [8]. Stone size and location influence the safety and success of PCNL. Xue et al. have assessed CROES data on 1,448 solitary nonstaghorn stones and found that large stones, particularly those bigger than 4 cm, were associated with significantly higher rates of fever and blood transfusion [9]. Opondod et al. have revealed that high-volume centers have lower transfusion rates, shorter length of stay, and better stone-free rates (SFRs) [10]. In this study, we used a large database from 2016 to 2019. This study was designed to determine the factors associated with blood transfusion after PCNL when unifying the sheath size and surgery methods in high-volume centers.

### 1.1. Patients and Methods

In this retrospective study, 665 patients who underwent PCNL at our department were included. Among the enrolled patients, 232 were female and 433 were male. Their mean age was 54.9 years (range 17–80 years). This study was approved by the Ethics Committee of Shanghai Xu-Hui Central Hospital (No. 2021-163).

### 1.2. Surgical Procedure

All procedures were performed under general anesthesia and in the prone position after retrograde ureteral catheterization. The selected calyx was accessed by Dr. G.J.M with ultrasound guidance using an 18-gauge needle. Then, a hard guidewire was inserted into the puncture needle. Then, the tract was dilated using serial dilators from an 8–20 F sheath. An 18 F nephroscope (Wolf) was used to inspect the sheath, and we used holmium laser to fragment stones with a power ranging from 40 to 90 watts. Every case was demanded to place an internal ureteral stent due to the suspicion of the presence of mobile residual stones. A 14 F nephrostomy tube was placed in the renal pelvis or the involved calyx for most patients.

The article "Factors Affecting Transfusion during Percutaneous Nephrolithotomy: A Retrospective Study of 665 Cases" was retracted in 2023. Reasons: signs of a paper mill; suspected computer-generated content; unreliable results or conclusions; lack of ethics approval or compliance.

All patients underwent urine routine and urinary bacterial culture examination before the operation. Urinary tract infection was defined as a white blood cell count of greater than 3+ in the urine.

When the bacterial culture is positive, antibiotics are used, and surgery is performed after the bacterial culture becomes negative.

Plain radiography of the kidneys, ureter, and bladder was performed on postoperative days 1–3 according to the state of the patient. For X-ray-negative stones, we used computed tomography (CT) for the postoperative follow-up. The nephrostomy tube was removed when there were no stone residual or clinically insignificant residual fragments (diameter less than 4 mm).

All patients were instructed to get the stent taken out 1 or 2 months after the surgery. If there were residual stones, the patients would undergo repeat PCNL, ureteroscopy, and shockwave lithotripsy (SWL). After that, all patients were evaluated using ultrasonography or noncontrast-enhanced CT 3–6 months after surgery. All patients were followed up for at least 1 year. During this period, they received follow-up calls or went to the clinic for regular check-ups.

PCNL was considered successful when the patient was stone-free or did not need any further intervention (clinically insignificant residual stone fragments).

### 1.3. Patients and Groups

Factors were categorized into three groups with relevance to individual variables, renal and stone factors, and surgical features. Individual variables consisted of sex; age; the presence of hypertension, diabetes mellitus, and urinary infection; serum creatinine level; preoperative hemoglobin; and the use of anticoagulant or antiplatelet medications. Renal and stone factors included previous surgery (i.e., open renal surgery, PCNL, ureteroscopic lithotripsy, or SWL treatment), abnormal anatomy (i.e., horseshoe kidney, double ureteropelvic malformation, and nephroptosis), stone side, stone burden, stone type, and degree of hydronephrosis. The kidney stone burden was estimated in terms of square area in millimeters by multiplying the length and width measured on preoperative plain abdominal radiographs. Stone types were categorized as staghorn calculi (partial or complete) and nonstaghorn stones. Hydronephrosis was graded as either nil/mild or moderate/severe using ultrasonographic criteria. Surgical features included the calyx of puncture and the number of access tracts. All factors were evaluated according to the presence of blood transfusion.

### 1.4. Statistical Analysis

The chi-square test, Fisher's exact test, and Student's *t*-test were used for univariate analyses. Multivariate binary logistic regression analysis was performed to investigate whether any parameter was significant with the univariate test. The results of the univariate and multivariate logistic regression analyses were provided in odds ratios (ORs) with 95% confidence intervals (CIs). *p*-values of less than 0.05 were used to denote statistical significance. The data were analyzed using Statistical Package for the Social Sciences, version 13.0.

The article "Factors Affecting Transfusion during Percutaneous Nephrolithotomy: A Retrospective Study of 665 Cases" was retracted in 2023. Reasons: signs of a paper mill; suspected computer-generated content; unreliable results or conclusions; lack of ethics approval or compliance.

## 2. Results

Severe bleeding, which needed transfusion, occurred in 23 of the 665 patients (3.5%). Twelve (1.9%) patients were treated with hyper-selective embolization. The average transfusion volume was 2.83 U RBC (range 1–6 U). For the transfusion group, the average hemoglobin amount before surgery was 114.6 g/L (range 63–138 g/L), the average hemoglobin amount at the first blood transfusion was 61.7 g/L (range 35–96 g/L), and the average hemoglobin loss was 52.9 g/L (Figure 1 shows the hemoglobin change in the patients). The distribution of cases with or without severe bleeding according to individual variables, renal and stone factors, and surgical features are shown in Tables 1–5, respectively.

## 3. Individual Variables

The mean age of the patients was 54.9 years (range 17–80 years). No significant correlation was found between sex, age, the presence of hypertension and diabetes mellitus, preoperative serum creatinine, and severe bleeding. However, preoperative hemoglobin had a strong correlation with severe bleeding (*p* < 0.001). Urinary infection increased the risk of bleeding in this study (*p* < 0.001) (Table 6).

Antiplatelet drugs were discontinued for 1 week before the operation for all patients, and for patients taking warfarin, the drug was discontinued 3 days before the operation, and heparin was used for bridging treatment. We found that the use of anticoagulants or antiplatelet medications has no significant correlation with blood transfusion following PCNL.

According to the logistic regression model, blood transfusion during PCNL was administered nine and 16 times in patients with anemic conditions and infection, respectively.

No significant difference in the transfusion rate was noted among factors including the position of the stone, stone size, and stone type. Among the factors of previous surgeries, only a history of open renal surgery was significantly correlated with severe bleeding. In our cases, the degree of hydronephrosis was also not correlated with severe bleeding following PCNL (*p* > 0.01).

In this study, 76 patients had received more than one access in the surgery. No significant correlation was noted between the number of access and severe bleeding or the calyx of entry. The total stone-free rate was 79.4% (528/665). For the transfusion group, their stone-free rate was 60.9% (14/23), which tended to be lower (*p* < 0.05) (Table 4).

The article "Factors Affecting Transfusion during Percutaneous Nephrolithotomy: A Retrospective Study of 665 Cases" was retracted in 2023. Reasons: signs of a paper mill; suspected computer-generated content; unreliable results or conclusions; lack of ethics approval or compliance.

## 4. Discussion

PCNL for renal calculi was first described by Fernstrom and Johansson in 1976 [1]. The complications of PCNL include fever, infection, bleeding necessitating transfusion, and bleeding necessitating super-selective angioembolization.

In this retrospective study, we studied 665 patients receiving PCNL at our center from 2016 to 2019. The risk of hemorrhagic complications requiring blood transfusion is associated with low preoperative hemoglobin levels, preoperative infection, and a history of open renal surgery. The OR was 9.3, 15.6, and 3.2, respectively.

Yamaguchi [8] and Christian [11] found that a larger tract size increases the risk of hemorrhage during PCNL. The transfusion rate varied from 1.1% to 12% when the tract size turned from 18 F to 30 F. In this study, we used a 20 F sheath and 18 F nephroscope to remove calculi. It was defined as a medium-size sheath [8]. The transfusion rate in this study was 3.5%. In three other studies involving more than 500 patients [12–14], a fixed tract size was used—30 F, 30 F, and 26–30 F, respectively—and the transfusion rate was 10.8%, 0.8%, and 12.3%, respectively; thus, bleeding may have increased due to the surgeries being performed at different centers rather than the size of the tract. Here we reviewed six studies (Table 7) [8, 12–16], which included more than 500 cases, and compared our data with those reported in the six aforementioned studies.

The number of access was thought to be associated with bleeding during PCNL. Nevertheless, studies had different results. It may be related to the proportions of multiple tracts of stone removal operations. Akman et al. [12] found that multiple access surgery increases the risk of bleeding by 2.7 times following PCNL (*p* <0.001). In that study, the percentage of multiple tract accesses was 22.7%. In another study, Soucy et al. [13] found no statistically significant difference in transfusion rates (0.7%–1.2%; *p* =0.24) between patients who were treated with a single tract and those needing multiple tracts. In their study, the percentage of multiple tract accesses was 16%. In this study, the percentage of multiple accesses was 11.5%. Few patients had multichannel puncture. Only 74 patients received two channels, and two patients had three channels, which would cause data bias. This is one of the limitations of this study.

Renal pelvic perforation was associated with bleeding in this study. A history of open surgery increases the risk of severe bleeding by three times. Patients with a history of open surgery may have a different kidney anatomy, which may increase the risk of bleeding at the puncture site. This result agrees with those reported by Christian [11]. In these six studies, only Akman [12] demonstrated that bleeding had no relationship with a history of surgery following PCNL.

The article "Factors Affecting Transfusion during Percutaneous Nephrolithotomy: A Retrospective Study of 665 Cases" was retracted in 2023. Reasons: signs of a paper mill; suspected computer-generated content; unreliable results or conclusions; lack of ethics approval or compliance.

This study found that preoperative hemoglobin levels were associated with blood transfusion, consistent with the results reported by Akman [12]. Among the patients who experienced bleeding in this study, 13 had preoperative anemia (average hemoglobin was 114.6 g/L), accounting for 56.5% with hemoglobin levels ranging from 63 g/L to 127 g/L. In the nontransfusion group, the preoperative anemia rate was 10.0%. The average hemoglobin loss was 52.9 g/L in the transfusion group. Among them, six patients had received a two-stage operation during one hospital stay. For them, the hemoglobin level before the second operation was 94 g/L. The average blood loss was 28.2 g/L. For patients who undergo a second-stage PCNL operation, if there is anemia before the operation, they will have a higher transfusion rate during PCNL.

Yamaguchi [8], Akman [12], and Srivastava [14] found that the stone load (size) was associated with bleeding during PCNL. Furthermore, operation time was associated with bleeding in the studies by Yamaguchi [8] and Akman [12]. Large stones often mean more puncture tracts and longer operation time. In this study, for staghorn calculi, the transfusion rate was 6.6%. Tracts were established by Dr. G.J.M in this study. He used an 18-gauge needle to access to the selected calyx with ultrasound guidance. The tract was dilated using serial dilators with an 8–20 F sheath. The overall process was completed within 5 min. With the updates in laser technology and better lithotripsy efficiency, the operation time can be greatly shortened. The operation time was not assessed in this study, which is a limitation of this study.

The caseload is also associated with bleeding during PCNL. In the CROES study, Opondo et al. [10] found that a high-volume center (>120 cases per year) usually has higher stone-free rates and lower complication rates. In studies reviewed previously, the transfusion rate was 5.24% and 3.4% (*p* < 0.001) in low- and high-volume centers, respectively.

A positive preoperative urine culture will increase bleeding complications following PCNL in both intraoperative and postoperative hematuria [17]. Despite antibiotic treatment before surgery, urine infection will increase the risk of severe bleeding in PCNL by 16 times. We had found that when infectious stones are seen during the establishment of access in the kidney, indwelling nephrostomy immediately for drainage and surgery stoppage are the best measures. Slightly increased operation time and water pressure will increase the risk of bleeding after PCNL.

The article "Factors Affecting Transfusion during Percutaneous Nephrolithotomy: A Retrospective Study of 665 Cases" was retracted in 2023. Reasons: signs of a paper mill; suspected computer-generated content; unreliable results or conclusions; lack of ethics approval or compliance.

We used plain abdominal radiography of the kidneys, ureters, and bladder or ultrasound for postoperative imaging. This test may result in false-negative results for stones. However, we used postoperative ultrasonography or CT to correct this bias. All patients were followed up for at least 1 year. The total stone-free rate was 79.4% (528/665). For the transfusion group, the SFR was 60.9% (14/23), and in the nontransfusion group, the SFR was 80.1% (514/642) (*p* = 0.031). The nontransfusion group was 2.5 times more likely to remove the stones than those who suffered serious bleeding after PCNL.

In this study, the blood transfusion rate was 3.5%. In previous studies involving more than 500 cases, the blood transfusion rate ranged from 0.8% to 12.3% [8, 12–16]. Therefore, our results were correlated with those of previous studies. Our center had a low transfusion rate compared with other centers. The reason may be attributed to the use of medium tract passage, ultrasound-guided puncture to save time, relatively few puncture tracts, and the application of high-power laser to fragment stones. A retrospective study involving 305 patients who underwent percutaneous nephrolithotomy reported a blood transfusion rate of 0%. Their experience is worth studying. Careful patient selection, accurate positioning, and the use of the best available instruments with well-trained urologists are necessary to avoid the complications associated with PCNL [6].

In this study, we have attempted to analyze PCNL in a high-volume center and previous case studies. Although it was a retrospective study, the obtained results demonstrated that PCNL is a safe procedure for an experienced surgeon. For a high-volume urolithiasis center, anemic conditions, infection before the surgery, and a history of open kidney surgery will significantly increase the risk of hemorrhagic complications following PCNL. The operation time was not assessed in this study as well as the time taken to achieve access into the desired calyx. This is a limitation of the study. Additionally, for the follow-up of stones, we used radiography of the kidneys, ureters, and bladder instead of CT. This may bring about a bias of a high postoperative success rate. Although we followed up the patients at least 1 year after surgery, there will definitely be data bias; however, overall, this study might have a ground-breaking interest for the readers regarding the significant factors affecting bleeding during PCNL.

The article "Factors Affecting Transfusion during Percutaneous Nephrolithotomy: A Retrospective Study of 665 Cases" was retracted in 2023. Reasons: signs of a paper mill; suspected computer-generated content; unreliable results or conclusions; lack of ethics approval or compliance.

## 5. Conclusion

For a high-volume center, anemic conditions, infection before surgery, and the history of open kidney surgery will significantly increase the risk of hemorrhagic complications following PCNL.

## Figures and Tables

**Figure 1:** Hemoglobin change in patients of transfusion.

**Table 1:** Patients' facts according to transfusion.

Parameters	Transfusion (+)% *n*	Transfusion (-)% *n*	*p* value
	23	642	
*Age (years)*	54.3 (18-73)	54.91(17-80)	0.954^a^
<50	30.4 (7)	31.0 (199)	
≥50	69.6 (16)	69.0 (443)	
*Sex*			0.379^a^
Female	43.5 (10)	34.6 (222)	
Male	56.5 (13)	65.4 (420)	

^a^Chi-square test.

**Table 2:** Individual parameters according to transfusion.

Parameters	Transfusion (+) % *n*	Transfusion (-) % *n*	*p* value
	23	642	
*Hypertension*			0.144^a^
(+)	43.5 (10)	32.4 (208)	
(-)	56.5 (13)	67.6 (434)	
*Diabetes mellitus*			0.756^b^
(+)	8.7 (2)	12.8 (82)	
(-)	91.3 (21)	87.2 (560)	
*Preoperative serum creatinine (umol/L)*			0.935^a^
<115	78.3 (18)	78.9(507)	
>115	21.7 (5)	24.1(135)	
*Anemia*			<0.001^b^
(+)	56.5 (13)	12.3(79)	
(-)	43.5 (10)	87.7(563)	
*Urinary infection*			<0.001^b^
(+)	69.6 (16)	12.8 (82)	
(-)	30.4 (7)	87.2 (560)	
*Use of anticoagulants or antiplatelet medications*			0.122^b^
(+)	8.7 (2)	3.0 (19)	
(-)	91.3 (21)	97.0 (623)	

^a^Chi-square test. ^b^Fisher's exact test.

**Table 3:** Renal factors according to transfusion.

Parameters	Transfusion (+) % *n*	Transfusion (-) % *n*	*p* value
	23	642	
*Grade of hydronephrosis*			0.104^a^
Nil or mild	17.4 (4)	33.6 (216)	
Moderate or severe	82.6 (19)	66.4 (426)	
*Abnormal anatomy*			0.067^b^
(+)	13.0 (3)	3.9 (25)	
(-)	87.0 (20)	96.1(617)	
*History of stone surgery*			
Open surgery			0.039^b^
(+)	21.7 (5)	8.1 (52)	
(-)	78.3 (18)	91.9 (590)	
PCNL			0.485^a^
(+)	17.4 (4)	23.7 (152)	
(-)	82.6 (19)	76.3 (490)	
URSL			0.433^a^
(+)	21.79 (5)	29.39 (188)	
(-)	78.3 (18)	70.7 (454)	
SWL			1^b^
(+)	8.7 (2)	10.4 (67)	
(-)	91.3 (21)	89.6 (575)	

^a^Chi-square test. ^b^Fisher's exact test.

**Table 4:** Stone factors according to transfusion.

Parameters	Transfusion (+) % *n*	Transfusion (-) % *n*	*p* value
	23	642	
*Side*			0.107^a^
Left	65.2 (15)	48.1 (309)	
Right	34.8 (8)	51.9 (333)	
*Stone size*	692.3 (40-2050 mm^2^)	708.5 (35-2980 mm^2^)	0.288^a^
<400mm^2^	47.8 (11)	32.4 (208)	
400-1000 mm^2^	34.8 (8)	41.7 (268)	
>1000m^2^	17.4 (4)	25.9 (166)	
*Stone type*			0.066^b^
Staghorn calculi	30.4 (7)	14.5 (93)	
Nonstaghorn calculi	69.6 (16)	85.5 (549)	

^a^Chi-square test. ^b^Fisher's exact test.

**Table 5:** Surgical factors according to transfusion.

Parameters	Transfusion (+) % *n*	Transfusion (-) % *n*	*p* value
	23	642	
*Access number*			1^b^
1	82.6 (19)	88.5(568)	
≥2	8.7(2)	11.5(74)	
*Calyx ox puncture*			
Upper	8.7(2)	5.5(35)	0.209^a^
Middle	65.2(15)	57.5(369)	
Low	26.1(6)	49.2(316)	
*Stone free rate*			
Residual	39.1 (9)	19.9(128)	0.031^a^
Clear	60.9 (14)	80.1 (514)	

^a^Chi-square test. ^b^Fisher's exact test.

The article "Factors Affecting Transfusion during Percutaneous Nephrolithotomy: A Retrospective Study of 665 Cases" was retracted in 2023. Reasons: signs of a paper mill; suspected computer-generated content; unreliable results or conclusions; lack of ethics approval or compliance.

**Table 6:** Outcomes of multivariate binary logistic regression analysis: factors affecting transfusion.

Factors	Significant	OR	95% CI
*Open surgery*	0.039		
(+)		3.152	1.13-8.83
(-)		1	
*Anemia*	<0.001		
(+)		9.265	3.93-21.84
(-)		1	
*Urinary infection*	<0.001		
(+)		15.61	6.23-39.10
(-)		1	

OR = odds ratio; CI = confidence interval.

**Table 7:** Studies on the factors associated with bleeding after PCNL of more than 500 cases.

Study	Yr	*N*	Transfusion rate %	Stone free rate %	Multiple tracts %	Tract size	Dilation methods	Factors associated with bleeding	Factors not associated with bleeding
Armitage et al. [10]	2012	1028	2.5	68	8	NA	Ballon, telescopic, serial	NA	Access obtainer, dilation methods, nephrostomy tube
Akman et al. [7]	2011	649	10.8	NA	22.7	30F	Ballon	Number of accesses, stone type, diabetes, preoperative hemoglobin level, operative time	Age, sex, BMI, stone opacity, stone side, grade of hydronephrosis, previous surgery, hypertension, creatinine level, surgeon experience, intraoperative complications
Yamaguchi et al. [5]	2011	5537	5.8	NA	NA	18F-34F	Ballon, telescopic, serial	Sheath size, operating time, stone load, caseload.	NA
Desai M et al. [11]	2011	1466 (staghorn)	9	56.9	NA	NA	Balloon, serial	NA	NA
		3869 (nonstaghorn)	4.5	82.5	NA	NA	Balloon, serial	NA	NA
Soucy F et al. [8]	2009	509	0.8	78	16	30F	Balloon, serial	Dilation methods	Number of accesses
Srivastava et al. [9]	2005	1854	12.3	NA	NA	26F-30F	Serial	Stone size	Number of punctures, creatinine level

## Data Availability

The data used to support the findings of this study are available from the corresponding author upon request.
